This article has been retracted.

# A facile sonochemical protocol for synthesis of 3-amino- and 4-amino-1,2,4-triazole derived Schiff bases as potential antibacterial agents

**DOI:** 10.1371/journal.pone.0229891

**Published:** 2020-06-04

**Authors:** Aeysha Sultan, Mian Habib Ur Rehman, Noreen Sajjad, Ali Irfan, Irfan Ullah, Muhammad Mustaqeem, Muhammad Saleem, Syeda Laila Rubab, Muhammad Rafiq, Muhammad Khalid, Katarzyna Kotwica-Mojzych, Mariusz Mojzych

**Affiliations:** 1 Division of Science and Technology, Department of Chemistry, University of Education, Lahore, Pakistan; 2 Department of Chemistry, University of Lahore, Lahore, Pakistan; 3 Department of Chemistry, University of Lahore Sargodha campus, Sargodha, Pakistan; 4 Department of Chemistry, University of Sargodha Sub-campus Bhakkar, Bhakkar, Pakistan; 5 Department of Physiology and Biochemistry, Cholistan University of Veterinary and Animal Sciences, Bahawalpur, Pakistan; 6 Department of Chemistry, Khwaja Ghulam Fareed University of Science and Technology, Rahimyar Khan, Pakistan; 7 Chair and Department of Histology, Embryology and Cytophisiology, Medical University of Lublin, (Collegium Medicum), Lublin, Poland; 8 Department of Chemistry, Siedlce University of Natural Sciences and Humanities, Siedlce, Poland; Aligarh Muslim University, INDIA

## Abstract

A facile method has been developed for the synthesis of Schiff bases derived from substituted and unsubstituted 3-amino- and 4-amino-1,2,4-triazoles. Condensation of the aminotrizoles with a variety of aromatic aldehydes afforded desired Schiff bases in excellent yields in 3–5 minutes of exposure to ultra-sound. The synthesized compounds were characterized by means of IR, ^1^HNMR and Mass spectrometry. The synthesized compounds were also screened for their antibacterial potential against Gram-negative (*Escherichia coli*, *Shigella sonnei*, *Pseudomonas aeruginosa* and *Salmonella typhi*) and two Gram-positive (*Staphylococcus aureus* and *Bacillus subtilis)* strains.

## Introduction

Schiff bases are the condensation products of primary amines and carbonyl compounds,[1] named after Hugo Schiff, who discovered them in 1864.[2] Schiff bases have been well documented for their wide spectrum potential as chemotherapeutic agents. The biological and chemical importance of the Schiff bases centers around the presence of azomethine group; it is the lone pair on nitrogen of azomethine that plays the key role.[3,4]

Schiff bases derivatives of aliphatic as well as aromatic aldehydes and ketones have been well reported; however, in general the stability of aliphatic aldehydes derived Schiff bases is quite inferior to that of aromatic aldehydes. The former being more prone to polymerization while the latter being more stable due to conjugation. [5]. Heterocyclic Schiff bases moiety is of special importance in medicinal chemistry and a lot of active research is being done on this pharmacophore. In addition to their importance in medicial chemistry, heterocyclic Schiff bases find promising potential applications as: sensors (optical and electrical), intermediates in organic reactions, dyes, pigments and as catalysts [6–9].

Hetereocyclic Schiff bases have been extensively documented for their potential as: antifungal [10,11], antibacterial [12,13], antiproliferative [14], anticoagulant [15], anti-inflammatory [16], and antiviral [17] agents. These heterocyclic Schiff bases have the added advantages of: ease of synthesis, electronic properties, higher solubility in organic solvents and most importantly for their potential role as chelating ligands in coordination chemistry [18].

The 1,2,4-triazole motif is a part of a large number of chemotherapeutic drugs [19,20] which are useful as: anti-inflammatory [21,22], anti-depressant, antiviral, antifungal, antimicrobial [23–27], anticancer properties [28–31], antitubercular [32–35] and analgesic [36], activities. Owing to the huge possibility of exploration of biologically active molecules containing this moety, a lot of work has been done on the synthesis of 1,2,4-triazole Schiff base derivatives [37–41].

A lot of work has been done to device strategies for the synthesis of Schiff bases; the most trivial method involves acid catalyzed condensation of an aldehyde (or ketone) with a primary amine under refluxing conditions. [42]. Due to attempts towards greener chemistry approaches, newer and unconventional methods are being explored in the field of synthetic chemistry. Various non-conventional methods employed in the synthesis of Schiff bases include: microwave assisted synthesis [43] and click chemistry [44–49].

The presented work is concerned with the synthesis of ultrasound assisted synthesis of Schiff bases derived from substituted and unsubstituted 3-amino and 4-amino-1,2,4-triazoles. The reaction outcome has also been compared with that of conventional method. Synthesized Schiff bases have also been evaluated for their antibacterial potential.

## Material and methods

The TLC was carried out on pre-coated silica gel (0.25 mm thick layer over Al sheet, Merck, Darmstadt, Germany) with fluorescent indicator. The spots were visualized under UV lamps (λ 365 and 254 nm) of 8 W power or KMnO_4_ dip and heating. The compounds were purified either on a glass column packed silica gel (0.6–0.2 mm, 60Å mesh size, Merck) or by crystallization. All solutions were concentrated under reduced pressure (25 mm of Hg) on a rotary evaporator (Laborota 4001, Heidolph, Germany) at 35–40°C. Melting points were determined using a MF-8 (Gallenkamp, Burladingen, Germany) instrument and are reported uncorrected. The IR-spectra are recorded on Prestige 21 spectrophotometer (Shimadzu, Japan) as KBr discs. The LREIMS are carried out on a Fisons Autospec Mass Spectrometer (VG, New Jersey, USA). The ^1^H (300, 400 and 500 MHz) and ^13^C-NMR (75 MHz) are recorded on AM-300, 400 and 500 MHz instruments (Bruker, Massachusetts, USA) in CDCl_3_ using TMS as internal standard. In spectroscopic data "A" means yield from conventional method and "B" means yield from sonochemical method.

### Representative conventional procedure for synthesis of triazole based Schiff bases

An equimolar mixture of amino-1,2,4-triazoles (10 mmol) and respective aldehydes (10 mmol) in methanol (40 mL) were refluxed for ~5 h. The completion of reaction was monitored by TLC. The reaction mixture was cooled to room temperature and filtered. After an hour, solid products were obtained from the solution. The precipitated products were recrystallized with hot ethanol.

### Representative sonochemical procedure for synthesis of triazole based Schiff bases

An equimolar mixture of amino-1,2,4-triazoles (1 mmol) and respective aldehydes (1 mmol) in methanol (4 mL) was subjected to ultra sound for ~5 minutes. The product started to precipitate within 3–4 minutes of sonochemical procedure. The completion of reaction was monitored by TLC. The solid product thus obtained was centrifuges and isolated by decantation of mother liquor. The isolated products were recrystallized with hot ethanol.

### 1-Phenyl-N-(4H-1,2,4-triazol-3-yl)methanimine, 6

Yield: 86% (A), 96% (B), M.p: 196°C. IR (KBr, cm^-1^): 3044 (N-H), 1634 (HC = N), 1592 (C = N), 1019 (N-N). ^1^H-NMR (DMSO-d6, δ): 8.34 (s, 1H, azomethine), 7.81–7.53 (m, 5H, Ar-H), 6.25 (s, 1H, N-CH = N). ^13^C-NMR (DMSO-d6, δ): 158.19 (HC = N), 153.83 (CH, triazole), 150.21 (C = N, triazole), 137.17 (C, Ar), 132.50 (C, Ar), 130.24 (CH, Ar), 127.38 (CH, Ar); EI MS: 178 [M] (67%), 177 [M-H]^+^ (100%). ESI MS (C_9_H_8_N_4_): 172.074905 (found); 172.074896 (calc).

### 2-(4H-1,2,4-Triazol-3-yl)iminomethylphenol, 7

Yield: 61% A), 96% (B); M.p: 264–265°C. IR (KBr, cm^-1^): 3188 (N-H), 3021 (O-H), 1624 (HC = N), 1605 (C = N), 1021 (N-N). ^1^H-NMR (DMSO-d6, δ): 8.78 (s, 1H, Azomethine), 7.84–7.13 (m, 4H, Ar-H), 6.25 (s, 1H, N-CH = N). ^13^C-NMR (DMSO-d6, δ): 159.14 (HC = N), 164.35 (C1, Ar), 153.23 (C5), 150.66 (C2), 134.11(CH, Ar), 121.13(CH, Ar), 116.08 (C, Ar). ESI MS (C_9_H_8_N_4_O): 188.069834 (found); 188.069811 (calc).

### 3-[(E)-4H-1,2,4-Triazol-3-yliminomethyl]naphthalen-2-ol, 8

Yield = 75% (A), 98% (B), M.p: 271°C. IR (KBr, cm^-1^): 3284 (O-H), 3089 (N-H), 1626 (HC = N), 1528 (C = N), 1023 (N-N). ^1^H-NMR (DMSO-d6, δ): 8.53 (s, 1H, azomethine), 8.27–7.35 (m, 6H, Ar-H), 9.24 (s, 1H, N-CH = N). ^13^C-NMR (DMSO-d6, δ): 159 (HC = N), 156 (C = C*-OH), 153 (N-CH = N), 150 ((N)2 -C = N), 140.1(1C, Ar), 128.15(1C, Ar), 126.08 (2C, Ar), 122.10 (2C, Ar), 115.93 (1C, Ar), 111.34 (2C, Ar). ESI MS (C_13_H_10_N_4_O): 238.086001 (found), 238.085461 (calc).

### 3-(4H-1,2,4-Triazol-3-yl)iminomethylbenzene-1,2-diol, 9

Yield = 58% (A), 92% (B). M.p: 282°C. IR (KBr, cm^-1^): 3273 (O-H), 3074 (N-H), 1623 (HC = N), 1601 (C = N), 1031 (N-N). ^1^H-NMR (DMSO-d6, δ): 3.14 (s, 2H, OH), 7.34–7.03 (m, 3H, Ar-H), 8.98 (s, 1H, azomethine), 9.23 (s, 1H, triazole); ^13^C-NMR (DMSO-d6, δ): 159.97 (HC = N), 154.23 (C, Ar), 153.24 (N-CH = N), 150.65 (C2, triazole), 148.56 (C, Ar), 128.61(C, Ar), 122.45 (C, Ar), 117.38 (CH, Ar). ESI MS (C_9_H_8_N_4_O_2_): 204.064681 (found); 204.064726 (calc).

### N,N-Dimethyl-4-[(E)-(4H-1,2,4-triazol-3-ylimino)methyl]aniline, 10

Yield: 79% (A), 99% (B); M.p: 203°C. IR (KBr, cm^-1^): 3092 (N-H), 1623 (HC = N), 1539 (C = N), 1032 (N-N). ^1^H-NMR (DMSO-d6, δ): 3.15 (s, 6H, (CH_3_)2-N), 6.23 (s, 1H, azomethine), 7.52–6.86 (m, 4H, Ar-H), 9.56 (s, 1H, HC = N); ^13^C-NMR (DMSO-d6, δ): 159.08 (HC = N), 153.02 (N-CH = N), 150.20 (C2, triazole), 132 (C, Ar), 127.06 (CH, Ar), 121.07 (C, Ar), 113.58 (CH, Ar), 43.33 [N(CH_3_)_2_]; ESI MS (C_9_H_8_N_4_O_2_): 215.117108 (found); 215.117095 (calc).

### 1-(4-Nitrophenyl)-N-(4H-1,2,4-triazol-3-yl)methanimine, 11

Yield: 67% (A), 97% (B); M.p: 269°C. IR (KBr, cm^-1^): 3102 (O-H), 3097 (N-H), 1638 (HC = N), 1595 (C = N), 1011 (N-N); ^1^H-NMR (DMSO-d6, δ): 6.23 (s, 1H, azomethine), 8.91–8.32 (m, 4H, Ar-H), 9.86 (s, 1H, HC = N); ^13^C-NMR (DMSO-d6, δ): 164.36 (HC = N), 153.83 (C5, triazole), 150.22 (C, Ar), 151.73 (CH, Ar), 148.06 (C, Ar), 127.66 (CH, Ar), 124.57 (C, Ar). ESI MS (C_9_H_7_N_5_O_2_): 217.06009 (found), 217.059975 (calc).

### 2-Ethoxy-4-[(E)-(4H-1,2,4-Triazol-3-ylimino)methyl]phenol, 12

Yield: 82% (A), 98% (B), M.p: 152°C. IR (KBr, cm^-1^): 3073 (N-H), 1633 (HC = N), 1580 (C = N), 1030 (N-N), ^1^H-NMR (DMSO-d6, δ): 1.15 (t, 3H, CH_3_), 4.16 (q, 2H, CH_2_), 7.53–6.96 (m, 3H, Ar-H), 8.38 (s, 1H, azomethone), 9.26 (s, 1H, CH, triazole), ^13^C NMR (DMSO–d_6_, δ): 161.18 (HC = N), 153.79 (N-CH = N), 150.26 (C2, triazole), 150.05 (CH, Ar), 148.00 (C, Ar), 132.50 (C, Ar), 125.06 (C, Ar), 117.33 (CH, Ar), 110.82 (C, Ar), 65.65 (CH2), 17.38 (CH_3_), ESI MS (C_11_H_12_N_4_O_2_): 232.09651 (found) 232.096026 (calc).

### 4-chloro-2-[(E)-(1H-1,2,4-triazol-3-ylimino)methyl]phenol, 13

Yield: 81% (A), 98% (B). Light-yellow. M.p: 222–224°C. IR (KBr, cm^-1^): 3273 (OH), 3184 (NH), 1636 (HC = N), 1610 (C = N), 1042 (N–N), 810 (C–Cl). ^1^H NMR (DMSO–d_6_, δ, ppm): 7.16 (d, 1H, *J* = 8.2 Hz, Ar-H), 7.46 (dd, 1H, *J* = 8.2, 2.4 Hz, Ar-H), 7.89 (d, 1H, *J* = 2.4 Hz, Ar-H), 8.44 (s, 1H, triazole C_9_–H), 9.40 (s, 1H, azomethine), 12.30 (s, 1H, OH), 13.98 (s, 1H, triazole NH). ^13^C NMR (DMSO–d_6_, δ, ppm): 118.1 (C_3_), 120.0 (C_1_), 129.2 (C_5_), 132.7 (C_6_), 134.2 (C_4_), 153.5 (C_9_), 156.9 (C_8_), 161.7 (C_7_), 162.9 (C_2_). Anal. Calcd. for C_9_H_7_ClN_4_O (222.63): C: 48.55; H: 3.17; N: 25.17; Cl: 15.92; Found: C: 48.32; H: 3.21; N: 25.08; Cl: 16.07%. ESI MS (C_9_H_7_N_4_OCl): 222.030893, 224.027952 (found, 3:1), 222.030839, 224.030839 (calc).

### 4-bromo-2-[(E)-(1H-1,2,4-triazol-3-ylimino)methyl]phenol, 14

Yield: 80% (A), 97% (B). Bright-yellow. M.p: 239–241°C. IR (KBr, cm^-1^): 3267 (OH), 3181 (NH), 1629 (HC = N), 1609 (C = N), 1027 (N–N). ^1^H NMR (DMSO–d_6_, δ, ppm): 7.18 (d, 1H, *J* = 8.2 Hz, Ar-H), 7.50 (dd, 1H, *J* = 8.2, 2.4 Hz, Ar-H), 8.00 (d, 1H, *J* = 2.4 Hz, Ar-H), 8.55 (s, 1H, triazole), 9.39 (s, 1H, azomethine), 12.51 (s, 1H, OH), 14.21 (s, 1H, triazole NH). ^13^C NMR (DMSO–d_6_, δ, ppm): 116.66 (CH_,_ Ar), 119.2 (CH, Ar), 121.4 (CH, Ar), 133.9 (C, Ar), 136.1 (C, Ar), 153.9 (CH = N), 156.98 (C = N), 161.75 (C2). Anal. Calcd. For C_9_H_7_BrN_4_O (267.08): C: 40.47; H: 2.64; N: 20.98; Br: 29.92; Found: C: 40.29; H: 2.56; N: 21.07; Br: 29.84%.

### 2-[(E)-{[5-(methylsulfanyl)-1H-1,2,4-triazol-3-yl]imino}methyl]phenol, 15

Yield: 72% (A), 90% (B). Light-yellow. M.p: 183–185°C. IR (KBr, cm^-1^): 3265 (OH), 3175 (NH), 1625 (HC = N), 1606 (C = N), 1030 (N–N). ^1^H NMR (DMSO–d_6_, δ, ppm): 2.62 (s, 3H, CH_3_), 6.95 (ddd, 1H, *J* = 7.90, 7.81, 2.4 Hz, Ar–H), 7.10 (dd, 1H, *J* = 7.84, 2.4 Hz, Ar–H), 7.44 (ddd, 1H, *J* = 7.90, 7.84, 2.35 Hz, Ar–H), 7.81 (dd, 1H, *J =* 7.81, 2.35 Hz, Ar–H), 9.37 (s, 1H, azomethine), 12.01 (s, 1H, OH), 14.12 (s, 1H, triazole NH). ^13^C NMR (DMSO–d_6_, δ, ppm): 13.9 (CH_3_), 116.7 (C, Ar), 119.3 (C, Ar), 131.7–134.5 (CH, Ar), 156.2 (C, Ar), 158.7 (C2_,_ triazole), 161.9 (C5_,_ triazole), 163.2 (CH = N). ESI MS (C_10_H_10_N_4_OS): 234.057598 (found), 234.057533 (calc).

### 4-chloro-2-[(E)-{[5-(methylsulfanyl)-1H-1,2,4-triazol-3-yl]imino}methyl]phenol, 16

Yield: 74% (A), 94% (B). Off-white. M.p: 214–215°C. IR (KBr, cm^-1^): 3281 (OH), 3183 (NH), 1634 (HC = N), 1610 (C = N), 1038 (N–N), 827 (C–Cl). ^1^H NMR (DMSO–d_6_, δ, ppm): 2.48 (s, CH_3_), 6.83 (d, 1H, *J* = 7.92 Hz, Ar-H), 7.30 (dd, 1H, *J* = 7.94, 2.5 Hz, Ar–H), 7.73 (d, *J* = 2.5 Hz, Ar–H), 9.14 (s, 1H, azomethine), 11.89 (s, 1H, OH), 13.98 (s, 1H, triazole NH). ^13^C NMR (DMSO–d_6_, δ, ppm): 13.9 (C, Ar), 118.7 (CH, Ar), 120.8(CH, Ar), 127.6 (CH, Ar), 131.8(C, Ar), 133.6 (C, Ar), 156.2 (C, Ar), 158.8 (C5, triazole), 162.1(C2, triazole), 163.2 (CH = N). Anal. Calcd. for C_10_H_9_N_4_SClO (268.72): C: 44.70; H: 3.38; N: 20.85; S: 11.93; Cl: 13.19; Found: C: 44.34; H: 3.24; N: 20.68; S: 12.04; Cl: 13.23%. ESI MS (C_10_H_9_N_4_SclO): 236.046505, 238.043610 (found, 3:1), 236.046489, 238.043539 (calc).

### 4-bromo-2-[(E)-{[5-(methylsulfanyl)-1H-1,2,4-triazol-3-yl]imino}methyl]phenol, 17

Yield: 76% (A), 97% (B). Greenish-yellow. M.p: 210–212°C. IR (KBr, cm^-1^): 3276 (OH), 3183 (NH), 1628 (HC = N), 1603 (C = N), 1024 (N–N). ^1^H NMR (DMSO–d_6_, δ): 2.60 (s, 3H, CH_3_), 6.95 (d, 1H, *J* = 7.89 Hz, Ar-H), 7.62 (dd, 1H, *J* = 7.89, 2.44 Hz, Ar-H), 8.00 (d, 1H, *J* = 2.44 Hz, Ar–H), 9.35 (s, 1H, azomethine), 12.12 (s, 1H, OH), 14.01 (s, 1H, triazole NH). ^13^C NMR (DMSO-d6, δ): 13.6 (CH_3_), 115.7 (C, Ar), 119.1 (CH, Ar), 121.4 (CH, Ar), 135.2 (CH, Ar), 136.3 (C, Ar), 156.4 (C, Ar), 158.1 (C5, triazole), 162.1 (C2, triazole), 163.4 (CH = N). Anal. Calcd. for C_10_H_9_BrN_4_OS(313.17): C: 38.35; H: 2.90; N: 17.89; S: 10.24; Br: 25.51; Found: C: 38.33; H: 2.63; N: 17.63; S: 10.19; Br: 25.64%.

### 2-[(E)-{[5-(methylsulfanyl)-1H-1,2,4-triazol-3-yl]imino}methyl]-4-nitrophenol, 18

Yield: 75% (A), 98% (B). Deep-yellow. M.p: 222–224°C. IR (KBr, cm^-1^): 3290 (OH), 3182 (NH), 1632 (HC = N), 1606 (C = N), 1360 (C–NO_2_), 1025 (N–N). ^1^H NMR (DMSO–d_6_, δ, ppm): 2.72 (s, 3H, CH_3_), 7.18 (d, 1H, *J* = 7.86 Hz, Ar-H), 8.30 (dd, 1H, *J* = 7.86, 2.45 Hz, Ar-H), 8.45 (d, 1H, *J* = 2.45 Hz, Ar-H), 9.40 (s, 1H, azomethine), 12.6 (s, 1H, OH), 14.10 (s, 1H, NH). ^13^C NMR (DMSO-D6, δ): 13.98 (CH_3_), 117.74 (C, Ar), 120.30 (CH, Ar), 125.58 (CH, Ar), 137.71 (C, Ar), 140.53 (CH, Ar), 156.27 (C, Ar), 158.44 (C2, triazole), 162.28 (C5, triazole), 163.34 (CH = N). Anal. Calcd. for C_10_H_9_N_5_SO_3_ (279.29): C: 43.01; H: 3.25; N: 25.08; S: 11.48; Found: C: 42.45; H: 2.98; N: 25.35; S: 11.64%.

### 2-{(E)-[(5-Amino-1H-1,2,4-triazol-3-yl)imino]methyl}-3-methoxyphenol, 19

Yield: 83% (A), 99% (B); colour (light yellow); M.p: 252–253°C; IR (KBr, cm^-1^): 3420 (OH), 3346 (NH_2_), 3187 (NH), 2910 (OCH_3_), 1628 (HC = N), 1595 (C = N, triazole), 1022 (N-N); ^1^H NMR (DMSO–d_6_, δ, ppm): 2.86 (s, 3H, OCH_3_), 6.98 (dd, 1H, *J* = 8.8, 8.9 Hz, Ar-H), 7.12 (d, 1H, J = *8*.*8* Hz, Ar-H), 7.53 (d, 1H, J = *8*.*9* Hz, Ar-H), 8.78 (s, 1H, azomethine), 10.22 (s, 1H, OH), 12.18 (s, 1H, NH); ^13^C NMR (DMSO-D6, δ): 55.4 (OCH_3_), 119.7 (C, Ar), 121.9 (CH, Ar), 124.2 (CH, Ar), 129.6 (CH, Ar), 150.0 (C, Ar), 151.0 (C, Ar), 156.6 (C2, triazole), 157.2 (C5, triazole), 162.3 (CH = N). LR EIMS (70eV) m/z (%): 233 ([M]^+^, 13), 218 (100), 202 (32), 177 (9), 171 (19), 164 (7), 150 (12), 134 (27), 123 (14), 104 (20), 77 (22); Anal. Calcd. for C_10_H_11_N_5_O_2_ (233.23): C 51.50, H 4.75, N 30.03, O 13.72; Found C 51.47, H 4.72, N, 29.98.

### 2-{(E)-[(5-Amino-1H-1,2,4-triazol-3-yl)imino]methyl}-5-chlorophenol, 20

Yield: 73% (A), 97% (B); colour (light yellow); M.p: 222–224°C; IR (KBr, cm^-1^): 3428 (OH), 3345 (NH_2_), 3192 (NH), 1636 (HC = N), 1606 (C = N, triazole), 1032 (N-N), 819 (C-Cl); ^1^H NMR (DMSO-d6, δ): 6.04 (s, 2H, NH_2_), 6.97 (d, 1H, J = *7*.*8* Hz, Ar-H), 7.48 (dd, 1H, J = *7*.*8*, *2*.*4* Hz, Ar-H), 7.84 (d, 1H, J = *2*.*4* Hz, Ar-H), 8.87 (s, 1H, azomethine), 10.26 (s, 1H, OH), 12.27 (s, 1H, NH); ^13^C NMR (DMSO-d6, δ): 120.27 (CH, Ar), 125.52 (CH, Ar), 131.72 (C, Ar), 133.13 (C, Ar), 156.12 (CH, Ar), 159.63 (C5, triazole), 160.33 (C2, triazole), 163.35 (CH = N); EIMS: [m/z, (%)]: 237, 235 [M]+ (100, 34), 221 (5), 205 (5), 181 (18), 166 (6), 154 (11), 131 (14), 127 (10), 111 (8), 75 (7); Anal. Calcd. for C_9_H_8_ClN_5_O (237.65): C 45.49, H 3.39, N 29.47; Found C 45.46, H 3.36, N 29.45.

### 2-{(E)-[(5-Amino-1H-1,2,4-triazol-3-yl)imino]methyl}- 5-bromophenol, 21

Yield: 77% (A), 95% (B); colour (light yellow); M.p: 227–229°C; IR (KBr, cm^-1^): 3424 (OH), 3343 (NH_2_), 3192 (NH), 1634 (HC = N), 1603 (C = N, triazole), 1027 (N-N), 564 (C-Br); ^1^H NMR (DMSO-d6, δ): 6.03 (s, 2H, NH_2_), 6.97 (d, 1H, *J* = 8.8 Hz, Ar-H), 7.58 (dd, 1H, *J* = 8.8, 2.4 Hz, Ar-H), 8.04 (d, 1H, *J* = 2.4 Hz, Ar-H), 8.83 (s, 1H, azomethine), 10.24 (s, 1H, OH), 12.25 (s, 1H, NH); ^13^C NMR (DMSO-d6): δ 119.78 (C, Ar), 121.34 (CH, Ar), 133.09 (CH, Ar), 136.53 (C, Ar), 156.12 (CH, Ar), 159.92 (C2, triazole), 158.78 (C5, triazole), 164.89 (CH = N); LR EIMS: [m/z, (%)]: 282, 284 [M]+ (100), 266 (13), 250 (7), 225 (20), 212 (8), 199 (26), 171 (5), 157 (9), 103 (14), 76 (11); Anal. Calcd. for C_9_H_8_BrN_5_O (282.09): C 38.32, H 2.86, N 24.83; Found C 38.28, H 2.84, N 24.81.

### 2-{(E)-[(5-Amino-1H-1,2,4-triazol-3-yl)imino]methyl}-5-nitrophenol, 22

Yield: 67% (A), 95 (B); dark yellow; M.p: 242–244°C; IR (KBr, cm^-1^): 3431 (OH), 3347 (NH_2_), 3199 (NH), 1648 (HC = N), 1617 (C = N, triazole), 1350 (NO_2_), 1054 (N-N); ^1^H NMR (DMSO-d6, δ): 6.07 (s, 2H, NH_2_), 7.19 (d, 1H, *J* = 8.7 Hz, Ar-H), 8.24 (dd, 1H, *J* = *8*.*7*, *2*.*3* Hz, Ar-H), 8.75 (d, 1H, J = *2*.*3* Hz, Ar-H), 9.83 (s, 1H, azomethine), 10.31 (s, 1H, OH), 12.30 (s, 1H, NH); ^13^C NMR (DMSO-d6): δ 120.8 (CH, Ar), 135.6 (CH, Ar), 140.7 (C, Ar), 156.1 (CH, Ar), 160.2 (C, Ar), 162.5 (C5, triazole), 166.1 (C2, triazole), 168.8 (CH = N); EIMS: [m/z, (%)]: 248 ([M]+, 22), 232 (100), 216 (20), 192 (31), 172 (5), 166 (19), 149 (22), 138 (11), 122 (14), 76 (10); Anal. Calcd. for C_9_H_8_N_6_O_3_ (248.19): C 43.55, H 3.25, N 33.86; Found C 43.52, H 3.22, N 33.83.

### 2-{(E)-[(5-Amino-1H-1,2,4-triazol-3-yl)imino]methyl}phenol, 23

Yield: 75% (**A**); 98% (**B**); colour (yellow); M.p: 181–183°C; IR (KBr, cm^-1^): 3420 (OH), 3350 (NH_2_), 3190 (NH), 1631 (HC = N), 1594 (C = N, triazole), 1025 (N-N); ^1^H-NMR (DMSO) δ: 6.01 (s, 2H, NH_2_), 6.98 (t, 1H, *J* = 8.4 Hz, Ar-H), 7.12 (d, 1H, *J* = *7*.*8* Hz, Ar-H), 7.41 (t, 1H, J = *7*.*4* Hz, Ar-H), 7.63 (d, 1H, J = *7*.*9* Hz, Ar-H), 8.81 (s, 1H, azomethine, Ar-H), 10.31 (s, 1H, OH), 12.22 (s, 1H, NH); ^13^C NMR (CDCl_3_): δ 117.7 (CH, Ar), 121.2 (CH, Ar), 130.3 (CH, Ar), 133.2 (C, Ar), 158.1 (C2, triazole), 159.8 (C5, triazole), 160.6 (CH = N),; LR EIMS: [m/z, (%)]: 203 ([M]^+^, 100), 186 (85), 172 (48), 161 (36), 147 (81), 132 (72), 120 (47), 104 (70), 91 (31), 77 (84); Anal. Calcd. for C_9_H_9_N_5_O (203.20): C 53.20, H 4.46, N 34.47; Found C 53.16, H 4.43, N 34.45.

### 4-[(4-Chloro-benzylidene)-amino]-5-(2,3,5-trichloro-phenyl)-4H-[1,2,4]triazole-3-thiol, 24

Yield: 46%, 92% (B), M.p: 148°C, IR (KBr, cm^-1^): 3082 (Ar-H), 3071 (NH/SH), 1617 (CH = N), 1594 (C = N), 1493 (C = C), 1019 (N-N). ^1^H-NMR (DMSO) δ: 7.33 (d, 2H, *J* = 8.7 Hz, 4-chlorophenyl), 7.53 (d, 2H, *J* = 8.4 Hz, Ar-H), 7.66 (d, 1H, *J* = 2.7 Hz, Ar-H), 7.91 (d, 1H, *J* = 2.4 Hz, Ar-H), 9.8 (s, 1H, azomethine), 14.29 (s, 1H, SH). LR EIMS: [m/z, (%)]: 418.8 (48), 417 (100), 415.2 (72), 387 (10), 335 (5), 307 (20), 289 (15), 281 (15), 232 (40).

### 4-[(4-Fluoro-benzylidene)-amino]-5-(2,3,5-trichloro-phenyl)-4H-[1,2,4]triazole-3-thiol, 25

Yield: 53% (A), 88% (B), M.p: 154°C; IR (KBr, cm^-1^): 3075 (NH), 3075 (Ar-H), 2910 (C-H), 1624 (HC = N), 1601 (C = N), 1612, 1486 (C = C), 1018 (N-N), 785 and 628 (C = Cl). ^1^H NMR (DMSO–d_6_, δ, ppm): 7.1–7.14 (t, 2H, *J* = 10.4 Hz, Ar-H), 7.474 (d, 1H, *J* = 2.7 Hz, Ar-H), and 7.68 (d, 1H, *J* = 2.4 Hz, Ar-H), 7.7–7.74 (m, 2H, Ar-H), 10.34 (s, 1H, N = CH), 11.29, (s, 1H, SH). LR EIMS: [m/z, (%)]: 404, 402, 400 [M^+^], (100, 100, 29), 403, 401, 399 [M-H] (100, 100, 30), 383 (20), 307 (30), 280 (50).

### N-(thiophen-2-ylmethylidene)-1H-1,2,4-triazol-3-amine, 26

Yield: 71% (A), 99% (B). Off-white. M.p: 172–174°C. IR (KBr, cm^-1^): 3175 (NH), 1628 (HC = N), 1611 (C = N), 1570, 1540 (C = C), 1020 (N–N), 960 (C–S). ^1^H NMR (DMSO–d_6_, δ, ppm): 7.24 (dd, 1H, *J* = 4.6, 4.0 Hz, thienyl–H), 7.8 (d, 1H, *J* = 4.0 Hz, thienyl–H), 7.89 (d, 1H, *J* = 4.6 Hz, thienyl–H), 8.25 (s, 1H, triazole–H), 9.30 (s, 1H, azomethine), 13.98 (s, 1H, triazole NH). ^13^C NMR (δ, ppm): 126.7 (CH, thienyl), 129.5 (CH, thienyl), 132.6 (C, thienyl), 153.5 (C5, triazole), 156.2 (C2, triazole), 159.0 (CH = N). Anal. Calcd. for C_7_H_6_N_4_S (178.21): C: 47.17; H: 3.39; N: 31.44; S: 17.99; Found: C: 47.30; H: 3.41; N: 31.35; S: 17.80%. ESI MS (C_7_H_6_N_4_S): 178.031359 (found) 178.031318 (calc).

### N-[(5-methylthiophen-2-yl)methylidene]-1H-1,2,4-triazol-3-amine, 27

Yield: 73% (A), 98% (B). Off-white. M.p: 168–170°C. IR (KBr, cm^-1^): 3185 (NH), 1632 (HC = N), 1612 (C = N), 1575, 1545 (C = C), 1020 (N–N), 965 (C–S). ^1^H NMR (DMSO–d_6_, δ, ppm): 2.5 (s, 3H, CH_3_), 6.96 (d, 1H, *J* = 3.0 Hz, thienyl-H), 7.60 (d, 1H, *J* = 3.0 Hz, thienyl–H), 8.20 (s, 1H, triazole–H), 9.20 (s, 1H, azomethine), 13.95 (s, 1H, triazole NH). ^13^C NMR (δ, ppm): 15.4 (CH_3_), 128.2 (C, thienyl), 130.9 (CH, thienyl), 137.6 (C, thienyl), 142.9 (CH, thienyl), 153.6 (C5 triazole), 156.5 (C2 triazole), 159.2 (CH = N). Anal. Calcd. for C_8_H_8_N_4_S (192.24): C: 49.98; H: 4.19; N: 29.14; S: 16.68; Found: C: 50.10; H: 4.10; N: 29.20; S: 16.61%. ESI MS (C_8_H_8_N_4_S): 192.047008 (found) 192.046968 (calc)

### N-[(3-methylthiophen-2-yl)methylidene]-1H-1,2,4-triazol-3-amine, 28

Yield: 74% (A), 96% (B). Light-brown. M.p: 171–173°C. IR (KBr, cm^-1^): 3180 (NH), 1626 (HC = N), 1610 (C = N), 1568, 1540 (C = C), 1020 (N–N), 970 (C–S). ^1^H NMR (DMSO–d_6_, δ, ppm): 2.46 (s, 3H, CH_3_), 7.06 (d, 1H, *J* = 4.5 Hz, thienyl–H), 7.79 (d, 1H, *J* = 4.5 Hz, thienyl–H), 8.20 (s, 1H, triazole–H), 9.29 (s, 1H, azomethine), 13.90 (s, 1H, triazole NH). ^13^C NMR (δ, ppm): 14.4 (CH_3_), 128.4 (C, thienyl), 129.3 (CH, thienyl), 132.9 (C, thienyl), 140.6 (CH, thienyl), 153.1 (C5 triazole), 156.8 (C2, triazole), 159.2 (CH = N). Anal. Calcd. for C_8_H_8_N_4_S (192.24): C: 49.98; H: 4.19; N: 29.14; S: 16.68; Found: C: 49.80; H: 4.00; N: 29.30; S: 16.57%. ESI MS (C_8_H_8_N_4_S): 192.047001 (found), 192.046968

### N-[(5-chlorothiophen-2-yl)methylidene]-1H-1,2,4-triazol-3-amine, 29

Yield: 59% (A), 91 (B). Light-brown. M.p: 178–180°C. IR (KBr, cm^-1^): 3190 (NH), 1629 (HC = N), 1610 (C = N), 1570, 1540 (C = C), 1020 (N–N), 970 (C–S), 820 (C–Cl). ^1^H NMR (DMSO–d_6_, δ, ppm): 7.39 (d, 1H, *J* = 3.5 Hz, thienyl–H), 7.70 (d, 1H, *J* = 3.5 Hz, thienyl–H), 8.5 (s, 1H, triazole–H), 9.24 (s, 1H, azomethine), 13.99 (s, 1H, triazole NH). ^13^C NMR (δ, ppm): 128.9 (CH, thienyl), 132.5 (CH, thienyl), 135.6 (C, thienyl), 146.2 (C, thienyl), 153.3 (C5, triazole), 156.9 (C2, triazole),159.3 (CH = N). Anal. Calcd. for C_7_H_5_ClN_4_S (212.66): C: 39.53; H: 2.37; N: 26.35; S: 15.08; Cl: 16.67; Found: C: 39.70; H: 2.34; N: 26.26; S: 15.13; Cl: 16.80%. ESI MS (C_7_H_5_ClN_4_S) = 211.992408, 213.989609 (found, 3:1), 211.992346, 213.989396 (calc).

### N-[(5-nitrothiophen-2-yl)methylidene]-1H-1,2,4-triazol-3-amine, 30

Yield: 79% (A), 89 (B). Brownish-green. M.p: 202–204°C. IR (KBr, cm^-1^): 3175 (NH), 1629 (HC = N), 1611 (C = N), 1560, 1540 (C = C), 1370 (C–NO_2_), 1020 (N–N), 980 (C–S). ^1^H NMR (DMSO–d_6_, δ, ppm): 7.72 (d, 1H, *J* = 4.1 Hz, thienyl–H), 7.87 (d, 1H, *J* = 4.1 Hz, thienyl-H), 8.30 (s, 1H, triazole–H), 9.27 (s, 1H, azomethine), 14.00 (s, 1H, NH). ^13^C NMR (δ, ppm): 129.9 (C, thienyl), 133.8 (CH, thienyl), 141.2 (CH, thienyl), 147.0 (C, thienyl), 153.6 (C5, triazole), 156.9 (C2, triazole), 159.1 (CH = N). Anal. Calcd. for C_7_H_5_N_5_SO_2_ (223.21): C: 37.67; H: 2.26; N: 31.38; S: 14.37; Found: C: 37.78; H: 2.34; N: 31.26; S: 14.45%. ESI MS (C_7_H_5_N_5_SO_2_): 223.016724 (found), 223.016397 (calc).

### N-[(E)-(4-bromothiophen-2-yl)methylidene]-1H-1,2,4-triazol-3-amine, 31

Yield: 69% (A), 98% (B). Off-white. M.p: 215–217°C. IR (KBr, cm^-1^): 3184 (NH), 1630 (HC = N), 1608 (C = N), 1570, 1545 (C = C), 1025 (N–N), 965 (C–S). ^1^H NMR (DMSO–d_6_, δ, ppm): 7.85 (d, 1H, *J* = 3.5 Hz, thienyl–H), 8.0 (d, 1H, *J* = 3.5 Hz, thienyl–H), 8.55 (s, 1H, triazole–H), 9.30 (s, 1H, azomethine), 14.00 (s, 1H, triazole NH). ^13^C NMR (δ, ppm): 116.7 (C_4_), 123.9 (C_5_), 125.2 (C_3_), 144.6 (C_2_), 153.4 (C_8_), 156.2 (C_7_), 159.5 (C_6_). Anal. Calcd. for C_7_H_5_N_4_SBr (257.11): C: 32.70; H: 1.96; N: 21.79; S: 12.47; Br: 31.08; Found: C: 33.06; H: 1.89; N: 22.10; S: 12.34; Br: 30.94%. ESI MS (C_7_H_5_N_4_SBr): 255.941909, 257.939824 (found, 1:1), 255.941829, 257.939783 (calc).

### N-[(E)-(3-methylfuran-2-yl)methylidene]-1H-1,2,4-triazol-3-amine, 32

Yield: 68% (A), 95% (B). Light-yellow. M.p: 106–108°C. IR (KBr, cm^-1^): 3190 (NH), 1630 (HC = N), 1609 (C = N), 1575, 1545 (C = C), 1090 (C–O), 1020 (N–N). ^1^H NMR (DMSO–d_6_, δ, ppm): 2.55 (s, 3H, CH_3_), 7.00 (d, 1H, *J* = 3.0 Hz, furanyl–H), 7.7 (d, 1H, *J* = 3.0 Hz, furanyl–H), 8.4 (s, 1H, triazole–H), 9.25 (s, 1H, azomethine), 13.95 (s, 1H, triazole, NH). ^13^C NMR (δ, ppm): 15.2 (CH_3_), 115.2 (CH, furanyl), 118.9 (CH, furanyl), 139.9 (C, furanyl), 144.6 (C, furanyl), 154.5 (C2, triazole), 156.5 (C2, triazole), 160.4 (CH = N). Anal. Calcd. for C_8_H_8_N_4_O (176.18): C: 54.54; H: 4.58; N: 31.80; Found: C: 54.75; H: 4.46; N: 31.97%. ESI MS (C_8_H_8_N_4_O): 176.069872 (found), 176.069811 (calc).

### N-[(E)-(5-chlorofuran-2-yl)methylidene]-1H-1,2,4-triazol-3-amine, 33

Yield: 68% (A), 97% (B). Light-yellow. M.p: 176–178°C. IR (KBr, cm^-1^): 3180 (NH), 1632 (HC = N), 1608 (C = N), 1565, 1546 (C = C), 1086 (C–O), 1025 (N–N), 830 (C–Cl). ^1^H NMR (DMSO–d_6_, δ, ppm): 7.38 (d, 1H, *J* = 3.5 Hz, furanyl–H), 7.49 (d, 1H, *J* = 3.5 Hz, furanyl–H), 8.5 (s, 1H, triazole–H), 8.90 (s, 1H, azomethine), 13.97 (s, 1H, triazole NH). ^13^C NMR (δ, ppm): 116.2 (CH, furanyl), 120.0 (CH, furanyl), 135.4 (C, furanyl), 142.6 (C, furanyl), 153.9 (C5, triazole), 155.5 (C2, triazole), 160.5 (CH = N). Anal. Calcd. for C_7_H_5_N_4_OCl (196.59): C: 42.77; H: 2.56; N: 28.50; Cl: 18.03; Found: C: 42.90; H: 2.43; N: 28.30; Cl: 18.11%. ESI MS (C_7_H_5_N_4_OCl): [M]^+^ = 196.015213, 198.012287 (found, 3:1), 196.015189, 198.012239.

### N-[(E)-(5-nitrofuran-2-yl)methylidene]-1H-1,2,4-triazol-3-amine, 34

Yield: 76% (A), 91% (A). Gray. M.p: 212–214°C. IR (KBr, cm^-1^): 3185 (NH), 1629 (HC = N), 1607 (C = N), 1570, 1548 (C = C), 1370 (C–NO_2_), 1080 (C–O), 1030 (N–N). ^1^H NMR (DMSO–d_6_, δ, ppm): 7.60 (d, 1H, *J* = 4.1 Hz, furanyl–H), 7.85 (d, 1H, *J* = 4.1 Hz, furanyl–H), 8.62 (s, 1H, triazole–H), 9.16 (s, 1H, azomethine), 14.20 (s, 1H, triazole NH). ^13^C NMR (δ, ppm): 120.6 (C, furanyl), 123.0 (C, furanyl), 143.2 (CH, furanyl), 147.0 (C, furanyl), 153.6 (C5, triazole), 156.7 (C2, triazole), 160.8 (CH = N). Anal. Calcd. for C_7_H_5_N_5_O_3_ (207.15): C: 40.59; H: 2.43; N: 33.81; Found: C: 40.23; H: 2.34; N: 34.20%. ESI MS (C_7_H_5_N_5_O_3_): 207.03991 (found), 207.03924 (calc).

### N-[(E)-1H-pyrrol-2-ylmethylidene]-1H-1,2,4-triazol-3-amine, 35

Yield: 61% (A), 92% (B),. Light-brown. M.p: 190–192°C. IR (KBr, cm^-1^): 3185 (NH), 3120 (NH), 1631 (HC = N), 1610 (C = N), 1570, 1540 (C = C), 1025 (N–N). ^1^H NMR (DMSO–d_6_, δ, ppm): 6.24 (dd, 1H, *J* = 4.6, 4.0 Hz, pyrrolyl–H), 6.86 (d, 1H, *J* = 4.0 Hz, pyrrolyl–H), 7.11 (d, 1H, *J* = 4.6 Hz, pyrrolyl–H), 8.30 (s, 1H, triazole–H), 8.89 (s, 1H, azomethine), 11.92 (s, 1H, pyrrolyl NH), 13.69 (s, 1H, triazole NH). ^13^C NMR (δ, ppm): 114.5 (CH, pyrrolyl), 116.6 (C, pyrrolyl), 120.7 (CH, pyrrolyl), 132.0 (C, pyrrolyl), 153.7 (C5, triazole), 155.8 (C2, triazole), 159.9 (CH = N). Anal. Calcd. for C_7_H_7_N_5_ (161.16): C: 52.17; H: 4.38; N: 43.45; Found: C: 52.39; H: 4.46; N: 43.72%. ESI MS (C_7_H_7_N_5_): 161.070185 (found), 161.070145 (calc).

### N-[(E)-(1-methyl-1H-pyrrol-2-yl)methylidene]-1H-1,2,4-triazol-3-amine, 36

Yield: 69% (A) 94% (B). Light-brown. M.p: 132–134°C. IR (KBr, cm^-1^): 3195 (NH), 1630 (HC = N), 1609 (C = N), 1024 (N–N). ^1^H NMR (DMSO–d_6_, δ, ppm): 3.30 (s, 3H, CH_3_), 6.19 (dd, 1H, *J* = 4.4, 4.1 Hz, pyrrolyl-H), 6.88 (d, 1H, *J* = 4.1 Hz, pyrrolyl–H), 7.18 (d, 1H, *J* = 4.4 Hz, pyrrolyl–H), 8.36 (s, 1H, triazole–H), 8.98 (s, 1H, azomethine), 13.62 (s, 1H, triazole NH). ^13^C NMR (δ, ppm): 31.2 (CH_3_), 113.6 (C, pyrrolyl), 117.8 (C, pyrrolyl), 122.5 (CH, pyrrolyl), 130.3 (CH, pyrrolyl), 153.6 (C5, triazole), 155.8 (C2, triazole), 159.4 (CH = N). Anal. Calcd. for C_8_H_9_N_5_ (175.19): C: 54.85; H: 5.18; N: 39.98; Found: C: 54.39; H: 5.27; N: 40.14%. ESI MS: (C_8_H_9_N_5_): 175.085816 (found), 175.085795 (calc).

## Results and discussion

For the synthesis of 1,2,4-triazole based Schiff bases, variously substituted and unsubstituted 3-amino and 4-amino-1,2,4-triazoles were employed. Condensation of these aminotriazoles with various aromatic aldehydes under ultrasound conditions would afford the desired Schiff bases (S1 File). For comparison purpose, the conventional method of synthesis of Schiff bases was also employed in parallel to ultrasound assisted synthesis.

### S1 File. Synthesis of target molecules

The conventional method involved refluxing the amine and aldehyde in ethanol for 4–5 hours. Upon cooling the reaction mixture at ambient temperature (and / or in ice bath under certain cases) led to the precipitation of the Schiff bases as solid products. In some cases the precipitates of the products were formed even during reaction process.

When the reaction was carried out in the presence of aq. HCl, a decrease in product yield was observed. Same was the case with acetic acid catalysed reaction. It is believed that the amino group of the triazole system is sufficiently nucleophilic to require any catalyst for the reaction. Furthermore, the use of acid catalysts tends to protonate and thereby reduces the nucleophilicity of the N of amino group. Conversely the reaction worked well in the absence of any catalyst.

The ultrasound mediated reaction was carried out by placing the ingredients of the reaction in a screw cap tube which was then placed in a sonicator. Subjecting the reaction contents to ultrasound resulted in immediate formation of product. The progress of reaction was monitored after every minute by means of TLC. The disappearance of both of the reactants on TLC was considered the completion of reaction. Majority of reactions got completed in 3 minutes and some took 4 minutes for completion.

The purity of the synthesized compounds was checked by TLC using a EtoAc/*n*-hexane (1:2) as mobile phase. All of the synthesized Schiff bases were soluble in DMSO, DMF while were soluble upon heating in methyl alcohol and ethyl alcohol. All products were stable to air as well. The synthesized compounds were characterized by means of FTIR, ^1^H NMR, ^13^C NMR and mass spectrometry.

The disappearance of the aldehydic carbonyl group as well as the stretching frequency corresponding to NH_2_ group of the triazole and appearance of characteristic azomethine (imine) absorption signal at 1580–1630 cm^-1^ in IR spectrum further strengthened the evidence of success of the reaction. In case of imines derived from 3,5-diamino-1,2,4-triazoles, the products exhibited an NH_2_ signal that appeared from 3343–3350 cm^-1^. In case of Schiff bases derived from 3-amino-1,2,4-trizoles and 4-amino-1,2,4-trizoles, the N-H of triazole appears 3187–3199 cm-1 (Fig 1).

**Fig 1:** 

The ^1^H NMR of the synthesized products exhibited presence of imine (CH = N) proton at 8.78–8.93 ppm. The appearance of the azomethine (aka imine) proton confirms the successful condensation and hence the formation of desired product.

The characteristic absorption frequencies and chemical shift values of azomethine proton of the Schiff bases are tabulated in Table 1.

**Table 1:** Melting points and characteristic spectroscopic/spectrometric signals of synthesized Schiff bases.

Compound No.	R^5^	Ar		M.P (C)		FTIR (absorption frequencies in cm^-1^)			NMR (chemical shift in ppm)		[M]+
				azomethine str	C = N str	N-N str	CH = N		CH = N		
**6**	H	Ph	196	1632	1590	1021	9.24		158.17		-
**7**	H	2-OHPh	263–264	1622	1604	1022	9.24		159.13		-
**8**	H	2-OHnaph	271	1626	1528	1023	9.24		159.00		-
**9**	H	3,4-(OH)_2_Ph	182	1622	1602	1030	8.99		159.98		-
**10**	H	4-(NMe_2_)Ph	203	1621	1540	1029	9.55		159.00		-
**11**	H	4-(NO_2_)Ph	269	1636	1596	1014	9.85		164.37		-
**12**	H	3-OEt,4-OHPh	151	1628	1572	1025	9.24		161.17		-
**13**	H	2-OH,5-ClPh	222–224	1631	1608	1030	9.40		161.67		222, 224 (3:1)
**14**	H	2-OH,5-BrPh	239–241	1632	1610	1028	9.39		161.75		266,268 (1:1)
**15**	SMe	2-OHPh	183–185	1625	1606	1030	9.35		161.93		234.29
**16**	SMe	2-OH,5-ClPh	214–215	1630	1607	1030	9.15		162.11		268, 270 (3:1)
**17**	SMe	2-OH,5-BrPh	210–212	1627	1605	1025	9.35		162.13		312.17,314.21 (1:1)
**18**	SMe	2-OH,5-NO_2_Ph	222–224	1632	1606	1025	9.40		162.28		279.29
**19**	NH_2_	2-OH,6-OMePh	252–253	1628	1595	1022	8.78		157.19		233
**20**	NH_2_	2-OH,4-ClPh	222–224	1636	1606	1032	8.87		160.33		235, 237 (3:1)
**21**	NH_2_	2-OH,4-BrPh	227–229	1634	1603	1027	8.83		158.78		282, 284 (1:1)
**22**	NH_2_	2-OH,4-NO_2_Ph	242–244	1648	1617	1054	9.83		166.05		248
**23**	NH_2_	2-OHPh	181–183	1631	1594	1025	8.81		160.63		203
**Compound No**			X		M.P (C)	FTIR (absorption frequencies in cm^-1^)			NMR (chemical shift in ppm)		[M]+
						azomethine str	C = N str	N-N str	C**H** = N	**C**H = N	
**24**			Cl		142	1617	1594	1019	9.80	-	418, 420 (3:1)
**25**			F		158	1624	1601	1018	10.34	-	401
Compound No.	X	R^3’^	R^4’^	R^5’^	M.P (C)	FTIR (absorption frequencies in cm^-1^)			NMR (chemical shift in ppm)		[M]+ (amu)
						azomethine str	C = N str	N-N str	C**H** = N	**C**H = N	
**26**	S	H	H	H	172–174	1628	1611	1020	9.30	156.0	178.21
**27**	S	H	H	Me	168–170	1632	1612	1020	9.20	156.5	192.24
**28**	S	Me	H	H	171–173	1626	1610	1020	9.29	156.8	192.00
**29**	S	H	H	Cl	178–180	1629	1610	1020	9.24	156.9	212.66, 214.80 (3:1)
**30**	S	H	H	NO_2_	202–204	1629	1611	1020	9.27	156.9	223.21
**31**	S	H	Br	H	215–217	1630	1608	1025	9.30	156.2	255.00, 257.18 (1:1)
**32**	0	Me	H	H	106–108	1630	1609	1090	9.25	156.5	176.18
**33**	0	H	H	Cl	176–178	1632	1608	1025	8.90	155.5	196.59, 198.64 (3:1)
**34**	0	H	H	NO_2_	212–214	1629	1607	1080	9.16	156.7	207.15
**35**	NH	H	H	H	190–192	1631	1610	1025	8.89	155.8	161.16
**36**	NMe	H	H	H	132–134	1630	1609	1024	8.97	159.3	175.19

The appearance of [M]^+.^ in LR EIMS further confirmed the formation of Schiff bases. The fragmentation pattern was consistent with that of desired product. The base peak was observed by loss of H as radical fragment in majority of cases (Fig 2).

**Fig 2:** The significantly higher yields of the product under ultra-sound mediated conditions may be attributed to the phenomenon of cavitations. The passing ultra-sound waves generate small bubbles in the reaction medium. These bubbles have energy trapped in them. These bubbles when combine form larger bubbles and hence large energy. When these bubbles rupture, the release energy which is sufficient enough to allow the reactant molecules overcome the energy barrier required for a specific reaction. The reaction under ultra-sound condition was significantly fast and all reactions afforded desired compounds as exclusive products in excellent yields.

### Antibacterial activities

Some representatives of the synthesized Schiff bases were evaluated for anti-bacterial activity. These compounds were tested for their effectiveness as antibacterial agents against gram positive (*S*. *aureus*, *B*. *subtilis*) and gram negative bacteria (*E*. *coli*, *S*. *flexneri*, *P*. *aeruginosa* and *S*. *typhi*). Imipenem was used as positive control in this study while filter paper disc dipped in 10% DMSO was used as negative control. In order to determine the antibacterial activity, 5 mg of each selected representatives were dissolved in 5 mL of DMSO to make up concentration of 1000 μg/mL. 0.1 mL of this solution was used for the determination of zone of inhibition. The zone of inhibition of different compounds was calculated in mm and mean ±SEM of triplicate data were calculated. The antibacterial activity was considered significant if the zone of inhibition was greater than 16 mm, the Schiff bases producing zone of 11–15 mm were considered moderately active while those with less than 10 mm zone were considered weakly active as antibacterial agents. The antibacterial activities of the selected Schiff bases are summarized in Table 2:

**Table 2:** Antibacterial activities of some selected Schiff bases.

Schiff base	Zone of inhibition (mm)					
	Bacterial strains					
	Gram positive	Gram negative			
	*S*. *aureus*	*B*. *subtilis*	*E*. *coli*	*S*. *flexneri*	*P*. *aeruginosa*	*S*. *typhi*
**6**	11	10	12	11	7	11
**8**	14	12	13	9	12	14
**10**	16	18	12	17	18	15
**11**	12	11	15	13	14	13
**15**	11	10	9	12	11	10
**16**	20	22	24	25	18	19
**17**	22	20	16	10	11	15
**19**	17	20	17	18	17	18
**20**	19	16	18	19	18	19
**22**	16	21	20	17	19	16
**23**	18	19	18	17	16	21
**24**	18	18	15	24	8	12
**25**	20	22	18	12	16	11
**26**	16	17	19	16	22	22
**27**	8	6	12	11	11	13
**28**	6	8	6	6	10	11
**29**	14	12	16	18	15	15
**30**	6	8	10	11	11	15
**31**	22	24	21	19	19	21
**35**	12	15	13	10	9	15
**36**	12	10	8	10	11	15
**Imipenem**	31	37	30	33	27	31

Establishing Structure activity relationship (SAR) from the zone of inhibition data is difficult however, some generalizations can be made. In case of 3-amino trizole derived Schiff bases, the presence of a bulky +R group promotes antibacterial activity while presence of a–R group decreases the activity (see entry 10 & 11, Table 2). Presence of a hydroxyl at *ortho* position of the benzene ring does not give any significant activity unless there is a +R group at position 5 of 6 of the aromatic ring. Presence of an SMe and /or NH_2_ group at C5 of the triazole ring promotes antibacterial activity. Any substituent present of C3 of aromatic ring has no influence on antibacterial activity. The 4-aminotriazole derived imines showed significant activity which may be attributed to presence of Cl and F. however, presence of a F atom at 4-position of the benzene ring gave more broader and efficient response than Cl atom at the same position; the later gave significant response against Gram positive bacteria. Among the schiff base derived from heterocyclic aldehydes, thienyl moiety exhibited better response than its oxygen and nitrogen counterparts. Again the presence of a halogen atom resulted in better activity. Since these studies were of preliminary nature, therefore further structure activity relationship studies require extensive exploration of the compounds.

## Conclusion

A series of 30 Schiff bases was synthesized by employing ultra-sound from sonicator as energy sourse. For comparison purpose, a conventional setup was also used. It was observed that former method afforded products with higher yields (88–99%) and higher purity in less time (almost 5 minutes). The yields of conventional method were significantly lower and took almost 5 hours for completion. These results are encouraging enough to explore the ultrasound mediated synthetic protocol for synthesis of other compounds of medicinal interests as well. some selective Schiff bases were subjected to preliminary antibacterial screening against Gram positive and Gram negative bacteria; the results exhibited promising results. The compounds that yielded good results will be further evaluated for their toxicology, MIC and MBC profile.

## Supporting information

S1 File Scheme 1. (CDX)

S1 Data (CDX)
